The article "Ammonia Scavenger Restores Liver and Muscle Injury in a Mouse Model of Non-alcoholic Steatohepatitis With Sarcopenic Obesity" was retracted in 2025. Reasons: plagiarism; overlap with other authors' work.

# Ammonia Scavenger Restores Liver and Muscle Injury in a Mouse Model of Non-alcoholic Steatohepatitis With Sarcopenic Obesity

**DOI:** 10.3389/fnut.2022.808497

**Published:** 2022-03-17

**Authors:** Zi-Xuan Wang, Meng-Yu Wang, Rui-Xu Yang, Ze-Hua Zhao, Feng-Zhi Xin, Yu Li, Tian-Yi Ren, Jian-Gao Fan

**Affiliations:** ^1^Department of Gastroenterology, Center for Fatty Liver, Xinhua Hospital Affiliated to Shanghai Jiao Tong University School of Medicine, Shanghai, China; ^2^Department of Hepatology, Qilu Hospital of Shandong University, Jinan, China; ^3^Chinese Academy of Science (CAS) Key Laboratory of Nutrition, Metabolism and Food Safety, Shanghai Institute of Nutrition and Health, University of Chinese Academy of Sciences, Chinese Academy of Sciences, Shanghai, China; ^4^Shanghai Key Lab of Pediatric Gastroenterology and Nutrition, Shanghai, China

**Keywords:** sarcopenia, obesity, ammonia, L-ornithine L-aspartate, steatohepatitis

## Abstract

Recent studies have revealed that sarcopenia is closely associated with obesity and non-alcoholic steatohepatitis (NASH). However, few attempted to explore the cause-and-effect relationship between sarcopenic obesity and NASH. In this study, we investigated muscular alterations in a rodent NASH model to elucidate their intrinsic relations and explore the potential therapeutic target. Forty-six 8-week-old and twenty 42-week-old male C57BL/6 mice (defined as young and middle-aged mice, respectively) were fed with a high-fat diet (HFD) for 12 or 20 weeks. A subset of young mice was subjected to ammonia lowering treatment by L-ornithine L-aspartate (LOLA). We examined body composition and muscle strength by nuclear magnetic resonance and grip strength meter, respectively. At the end of the 12th week, all HFD-fed mice developed typical steatohepatitis. Meanwhile, sarcopenia occurred in HFD-fed middle-aged mice, whereas young mice only demonstrated decreased grip strength. Until the end of week 20, young mice in the HFD group exhibited significant sarcopenia and obesity phenotypes, including decreased lean body mass and grip strength, and increased body fat mass and percentage body fat. Additionally, plasma ammonia level was markedly increased in HFD-fed mice of both ages at week 20. Plasma ammonia level was negatively associated with muscle strength and myofiber diameter in young mice. LOLA can significantly reduce plasma levels of ammonia, alanine aminotransaminase, aspartate aminotransaminase, and cholesterol in mice fed an HFD. Hepatic infiltration of inflammatory cells and collagen deposition area were significantly decreased in HFD group by LOLA treatment. Meanwhile, LOLA significantly increased lean body mass, grip strength, and average muscle fiber diameter of HFD-fed mice. These findings suggest that the occurrence of NASH precedes sarcopenia in HFD mice, and the steatohepatitis-related hyperammonemia might contribute to the pathogenesis of sarcopenia. LOLA might be an effective drug for both steatohepatitis and sarcopenic obesity.

The article "Ammonia Scavenger Restores Liver and Muscle Injury in a Mouse Model of Non-alcoholic Steatohepatitis With Sarcopenic Obesity" was retracted in 2025. Reasons: plagiarism; overlap with other authors' work.

## Introduction

Non-alcoholic fatty liver disease (NAFLD) is a metabolic stress-related liver injury involving metabolic dysfunction and genetic susceptibility, and the disease spectrum covers non-alcoholic fatty liver, non-alcoholic steatohepatitis (NASH), liver fibrosis, cirrhosis, and even hepatocellular carcinoma (HCC) (1). Although obesity is a major risk factor for NAFLD and NASH, there is a proportion of NAFLD patients have a normal body mass index (BMI) (2). The term “non-obese” refers to individuals with a normal BMI or overweight, and nearly 40% of the NAFLD patients are non-obese (3). The risk of NASH and other metabolic diseases for non-obese patients is not lower than obese individuals, as they can also develop HCC and cardiovascular disease (4, 5). However, the pathogenesis of non-obese NAFLD remains unclear. One of many possible hypotheses would be that the existence of skeletal muscle loss weakens the sensitivity and specificity of BMI in the diagnosis of obesity. Therefore, approaches like dual-energy X-ray absorptiometry or magnetic resonance imaging (MRI) could do better in detecting the body composition of NAFLD patients and thus promptly assist screening of patients who complicated by occult obesity or sarcopenia (6).

The word “sarcopenia” was originally used to delineate aging-related decline of skeletal muscle mass and function. While in addition to aging, multiple factors have been linked with the development of sarcopenia, such as malnutrition, sedentary behavior, and chronic diseases (diabetes, chronic liver disease, etc.) (7). Previous studies have uncovered the close association between NAFLD and sarcopenia. The prevalence of sarcopenia gradually increases as NAFLD progresses (8). Vice versa, sarcopenia increases the risk of developing NASH or liver fibrosis in NAFLD patients and influences the mortality of cirrhosis (9, 10). Moreover, sarcopenia is not uncommon in non-obese individuals. Both muscular mass and strength in non-obese NAFLD patients were noted significantly lower compared with obese patients (11). Accordingly, it is essential for clinical workers to pay more attention to the assessment of skeletal muscle status of NAFLD patients and find an effective treatment to address both liver disease and sarcopenia. Regrettably, most clinical studies in this regard are cross-sectional studies. Although they revealed the potential link between NAFLD and sarcopenia, they failed to elucidate their causal relationship. Further animal studies are warranted to reveal the detailed relationship between the two diseases and provide new ideas for their treatment strategies.

The article "Ammonia Scavenger Restores Liver and Muscle Injury in a Mouse Model of Non-alcoholic Steatohepatitis With Sarcopenic Obesity" was retracted in 2025. Reasons: plagiarism; overlap with other authors' work.

Numerous potential mediators of liver-muscle axis have been proposed including decreased testosterone and growth hormone, ammonia, and endotoxemia (12–14). Among these, ammonia has been studied most extensively. Chronic liver diseases can lead to hyperammonemia which contributes to muscle depletion through diverse mechanism such as increasing the expression of myostatin, impairing bioenergetics in the muscle, and so forth (15). Due to the dysfunction of urea cycle, NAFLD also causes hyperammonemia and this alteration of ammonia metabolism will promote the development of liver fibrosis in NAFLD patients (16, 17). Given this, we hypothesized that ammonia lowering may be an effective means of treating liver and muscle injuries simultaneously in NAFLD. In this study, we investigated the detailed relationship between NAFLD and sarcopenia in a mouse model of high-fat diet (HFD)-induced steatohepatitis, and explored the therapeutic efficacy of ammonia scavenger L- ornithine L- aspartate (LOLA) for steatohepatitis and sarcopenic obesity in this model. These *in vivo* studies demonstrated that (1) long-term HFD feeding can establish a mouse model of NASH with sarcopenic obesity; (2) the occurrence of steatohepatitis precedes sarcopenia in this model; (3) LOLA can effectively alleviate HFD-induced steatohepatitis and sarcopenic obesity.

## Materials and Methods

### Animal Experiment

Twenty-eight 8-week-old and twenty 42-week-old male mice (C57BL/6 background) were purchased from Shanghai Model Organisms Center, Inc. (Shanghai, China), and were named young and middle-aged group, respectively. Mice were randomized to receive either a normal chow diet or a high-fat high-cholesterol diet (HFD, 33% calories from fat, 50% carbohydrates, 17% protein, and 2% cholesterol; TrophicDiet, Nantong, China) for 20 weeks. Mice from the different diet condition and age groups were randomly sacrificed at the end of the 12th week. Subsequently, all mice were treated with normal saline by gavage for 8 weeks and were sacrificed at the end of the 20th week. The other eighteen 8-week-old male mice were fed on a normal chow diet or HFD for 12 weeks. Then, these mice were treated with LOLA (2g/kg/day, a generous gift from QR Pharmaceuticals, Wuhan, China) by gavage once daily for 8 weeks. All mice were housed at a controlled temperature and maintained at 12/12-h day-night cycle. All animal experiment protocols were approved by the Institutional Animal Care and Use Committee of Xinhua Hospital Affiliated to Shanghai Jiao Tong University School of Medicine, and the experiment flow chart is shown in Supplementary Figure 1.

The article "Ammonia Scavenger Restores Liver and Muscle Injury in a Mouse Model of Non-alcoholic Steatohepatitis With Sarcopenic Obesity" was retracted in 2025. Reasons: plagiarism; overlap with other authors' work.

### Forelimb Grip Strength Test

Mice's forelimb grip strength was measured by a grip strength meter (Bioseb, Model: BIO-GS3, France) 24 h before body composition examination. The procedure was performed following the manufacturer's instruction. Briefly, the strength meter was placed on the horizontal plane and reset to 0 g after stabilization. When a mouse grasped the bar, the mouse's tail was slowly pulled back at a constant speed by an operator and the peak pull value was recorded on a digital force transducer. We performed 3 consecutive measurements per mouse at 5-min intervals. The average of three measurements was taken as the final strength value. Measurements were repeated by 2 operators to ensure the reliability and reproducibility of the data.

### Body Composition Examination

Before mice were sacrificed, we measured the body composition of mice by nuclear magnetic resonance (NMR; Minispec LF50, Bruker Optics, Germany) after anesthesia. We collected fat mass, lean body mass, and body water over the entire body range using NMR. The percentage body fat and lean body mass of mice was calculated as the ratio between the value of the total amount of fat mass or lean body mass and the bodyweight (BW) of mice. The data were represented as Fat mass/BW and lean mass/BW.

### Plasma and Liver Biochemical Indexes Measurements

Plasma sample was obtained by centrifugation at 3,000 rpm for 15 min at 4°C. Plasma ammonia level was assayed by using the ammonia assay kit (Sigma-Aldrich AA0100) according to the manufacturer's protocol. Briefly, 100 μl of plasma sample was mixed with 1 ml of ammonia assay reagent and incubated at room temperature for 5 min. Subsequently, 10 μl of glutamate dehydrogenase solution was added and the absorbance was read at 340 nm after 5 min incubation. The standard curves were plotted, and the concentration of plasma ammonia was calculated according to the standard curve.

Alanine aminotransaminase (ALT) assay kit (cat. 3050280) and aspartate aminotransaminase (AST) assay kit (cat. 3040280) were purchased from Shensuo UNF (Shanghai, China). Plasma ALT and AST levels were measured according to the manufacturers protocol. Total cholesterol kit (cat. 104) purchased from Shensuo UNF (Shanghai, China) was used for the measurement of plasma lipid. After weighing the wet weight of liver and calculating the liver index (liver weight/body weight), liver homogenates were prepared immediately for subsequent experiment. Liver triglyceride and cholesterol level were assayed by a triglyceride assay kit (cat. E1013; Applygen Technologies Inc., Beijing, China) and a total cholesterol assay kit (cat. E1015; Applygen Technologies Inc., Beijing, China). Measurements of liver lipids were normalized to total protein of liver.

The article "Ammonia Scavenger Restores Liver and Muscle Injury in a Mouse Model of Non-alcoholic Steatohepatitis With Sarcopenic Obesity" was retracted in 2025. Reasons: plagiarism; overlap with other authors' work.

### Histological Evaluation of Liver and Muscle

The right lobe of the liver and the quadriceps muscle were isolated and fixed in 10% phosphate-buffered formalin acetate at 4°C and then embedded in paraffin wax. Paraffin sections were cut into 5 μm and stained with hematoxylin and eosin (HE) as previously described (18). Sirius Red staining of the liver sections was carried out using the picrosirius red staining solution according to the standard methods in routine pathology. The area of fibrosis in the liver was determined by detecting collagen deposition (red) using ImageJ software (National Institutes of Health, Bethesda, MD). Immunohistochemistry staining of liver sections was performed as previously describe (19). Following rabbit polyclonal antibodies were used as a primary antibody: anti-CD68, anti-F4/80, anti-myeloperoxidase (MPO) and anti-α-smooth muscle actin (αSMA). All primary antibodies were purchased from Servicebio Technology Co., Ltd (Wuhan, China). Quantification of staining intensity was done using the Image J software. Myofiber diameter was measured by ImageJ software. For each muscle section, the diameter of at least 30 myofibers was measured at 20x magnification, and the mean diameter was calculated.

### RNA Isolation and Quantitative RT-PCR Analysis of the Liver

Liver tissues were homogenized in TRIzol reagent (Life Technologies, Carlsbad, CA, USA). RNA was reverse transcribed using the HiScript II Q RT SuperMix for qPCR Kit (Vazyme, Nanjing, China). The resulting cDNA was subjected to real-time PCR with gene-specific primers in the presence of SYBR Green PCR master mix (Applied Biosystems) using StepOnePlus Real-Time PCR System (Applied Biosystems) as described previously (20). The following quantitative RT-PCR primer sequences were used: CATTGCTGACAGGATGCAGAAGG (Forward) and TGCTGGAAGGTGGACAGTGAGG (Reverse) for mouse β-actin; GGAGCCATGGATTGCACATT (Forward) and GGCCCGGGAAGTCACTGT (Reverse) for mouse SREBP1c; GCTGCGGAAACTTCAGGAAAT (Forward) and AGAGACGTGTCACTCCTGGACTT (Reverse) for mouse FAS; TTCTTCTCTCACGTGGGTTG (Forward) and CGGGCTTGTAGTACCTCCTC (Reverse) for mouse SCD1; GGGCAGAGCAAGTCATCTTC (Forward) and CCTCTGGAAGCACTGAGGAC (Reverse) for mouse PPARα; CCAGGCTACAGTGGGACATT (Forward) and GAACTTGCCCATGTCCTTGT (Reverse) for mouse CPT1A; ATTTCACTTCCAAGGCTGCC (Forward) and CTGGTCCTGGTCATCTCTCC (Reverse) for mouse TNFα; AGTTGCCTTCTTGGGACTGA (Forward) and TCCACGATTTCCCAGAGAAC (Reverse) for mouse IL-6; TTAAAAACCTGGATCGGAACCAA (Forward) and GCATTAGCTTCAGATTTACGGGT (Reverse) for mouse CCL2; AGCACATGTGGTGAATCCAA (Forward) and TGCCATCATAAAGGAGCCA (Reverse) for mouse CCR2; TGCTTCCTCCTCCTCCTTTG (Forward) and GAAGTACTGCCGTTTTCCCC (Reverse) for mouse αSMA; CCTGCAAGACCATCGACATG (Forward) and GCGAGCCTTAGTTTGGACAG (Reverse) for mouse TGFβ; CCAGCAAACAAAGGCAATGC (Forward) and GGTGCTGGGTAGGGAAGTAG (Reverse) for mouse COL1α1; CAACTCAGCTCGCCTTCATG (Forward) and CTCATCCAGGTACGCAATGC (Reverse) for mouse COL1α2.

The article "Ammonia Scavenger Restores Liver and Muscle Injury in a Mouse Model of Non-alcoholic Steatohepatitis With Sarcopenic Obesity" was retracted in 2025. Reasons: plagiarism; overlap with other authors' work.

### Working Definition

In this study, some working definitions were formulated according to the related literature. NASH was diagnosed when steatosis, lobular inflammation, and hepatocyte ballooning were concomitantly present (21). The histopathological scoring of liver sections was evaluated based on the NAFLD activity score (NAS) (21). Briefly, steatosis was scored from 0 to 3 based on the quantities of lipid droplets (0: <5%; 1: 5–33%; 2: 33–66%; 3: >66%). Lobular inflammation was scored from 0 to 3 based on the number of inflammatory foci (0: none; 1: <2 foci per 20 ×; 2: 2–4 foci per 20 ×; 3: >4 foci per 20 ×). Hepatocyte ballooning was scored from 0 to 2 (0: none; 1: few balloon cells; 2: many cells/prominent ballooning). Obesity was defined as a significant increase in body weight or body fat mass. Sarcopenia was diagnosed when mice having the presence of both low muscle mass and strength (22). When mice fulfilled the criteria of both sarcopenia and obesity, it could be considered sarcopenic obesity (23).

### Statistical Analysis

Data were presented as mean ± the standard error of the mean (SEM). Comparisons between groups were performed using the Student's *t*-test for only two groups or using one-way ANOVA for more than two groups. The correlations between plasma ammonia level and other indexes were evaluated by Spearman's correlation. *P*-values of <0.05 were considered statistically significant. All statistical analyses were carried out using GraphPad Prism (version 8.0; GraphPad Software, San Diego, USA) and SPSS 21.0 (IBM SPSS, USA).

## Results

### Muscle Strength, but Not Muscle Mass, Was Decreased in Young Mice With HFD for 12 Weeks

At the end of week 12, all mice receiving the HFD feeding developed typical histopathological features of NASH, significantly increased NAS score and liver indexes (Figures 1A,B,D). Although steatohepatitis has been successfully induced, body weights of mice in the HFD-fed group did not increase significantly, but was similar to that in the chow-fed group (Figure 1C). The presentation of these NASH mice resembles the NAFLD patients who displayed a normal BMI. Using a body composition analyzer, we measured body composition of mice. Compared with the chow-fed group, the body fat mass and percentage body fat of middle-aged HFD-fed mice were significantly increased, while the lean body mass and grip strength were significantly reduced (Figures 1E–G). Nevertheless, such body composition alterations only appeared in the middle-aged mice. Even though the grip strength of HFD-fed young mice was significantly decreased in week 12, we observed no body composition changes as above (Figures 1E–G).

The article "Ammonia Scavenger Restores Liver and Muscle Injury in a Mouse Model of Non-alcoholic Steatohepatitis With Sarcopenic Obesity" was retracted in 2025. Reasons: plagiarism; overlap with other authors' work.

**Figure 1:** Twelve weeks HFD feeding induced steatohepatitis and decreased muscle strength in mice. 8-week-old and 42-week-old male C57BL/6 mice were fed with a high-fat diet (HFD) for 12 weeks, mice were sacrificed after the assessment of body composition and muscle strength, and liver and muscle tissues were harvested. **(A)** Representative hematoxylin and eosin staining of mice liver and **(B)** NAFLD activity score (*n* = 3–5) are shown (scale bar, 50μm). **(C)** Body weights and **(D)** Liver indexes were assessed in mice (*n* = 3–5). Body composition was measured by nuclear magnetic resonance (NMR), **(E)** Fat mass, Fat mass/bodyweight (BW), **(F)** Lean mass/BW are shown (*n* = 3–5). **(G)** Forelimb grip strength are detected (*n* = 8–29). The data are presented as the mean ± SEM, unpaired two-tailed Student's *t*-test. *P < 0.05, **P < 0.01, ***P < 0.001, ****P < 0.0001.

### Muscle Histology Was Unchanged After 12 Weeks of HFD Feeding

We next weighed the muscles and performed HE staining to evaluate histopathological changes in the muscle. As shown in Figure 2A, chow-fed young mice used as controls had a normal muscle weight. HFD-fed young mice had lower quadriceps weight and quadriceps weight to body weight ratio than chow-fed controls (Figures 2A,C). A similar trend was observed for gastrocnemius even if not statistically significant (Figures 2B,D; gastrocnemius weight *P* = 0.056; gastrocnemius/BW *P* = 0.055). The muscle weight of HFD-fed middle-aged mice did not show any change in either absolute value or ratio when compared to its chow-fed controls (Figures 2A,B–D). The percentage of muscles weight to body weight in the middle-aged mice was holistically smaller than in the young mice, and the difference reached statistical significance in the chow-fed group (Figures 2C,D). Nevertheless, there were no appreciable difference among histological appearance of muscle and myofiber diameters in each group (Figures 2E,F).

**Figure 2:** Muscle weight and histological changes of mice fed with HFD for 12 weeks. **(A)** Quadriceps and **(B)** gastrocnemius muscle weight in mice (*n* = 3–5). **(C)** Quadriceps weight or **(D)** gastrocnemius weight as a percentage of total body weight are calculated (*n* = 3–5). **(E)** Representative hematoxylin and eosin staining of quadriceps in mice (*n* = 3–5) are shown (scale bar, 50 μm). **(F)** Quantification of mean muscle fiber diameters was performed by Image J software (*n* = 3–5). The data are presented as the mean ± SEM, unpaired two-tailed Student's *t*-test. *P < 0.05, **P < 0.01.

The article "Ammonia Scavenger Restores Liver and Muscle Injury in a Mouse Model of Non-alcoholic Steatohepatitis With Sarcopenic Obesity" was retracted in 2025. Reasons: plagiarism; overlap with other authors' work.

### Twenty Weeks of HFD Feeding Induced Sarcopenic Obesity in Young Mice

By the end of the 20th week, liver histological features of HFD-fed mice were consistent with typical NASH manifestations (Figure 3A), and the NAS score and liver indexes of HFD-fed mice significantly increased compared with the chow-fed controls (Figures 3B,D). while there were still no significant differences in body weight between the chow-fed mice and the HFD-fed mice (Figure 3C). Compared with the chow-fed controls, HFD-fed young mice presented not only low grip strength (Figure 3G) in week 20, but also obvious body composition changes including increased body fat mass and percentage body fat, and decreased lean body mass (Figures 3E,F). The phenotypes of HFD-fed young mice fulfilled the definition of sarcopenic obesity in this study. HFD-fed mice in middle-aged group had the same muscle phenotypes as young mice, and the grip strength of them was much lower than that of young mice (Figure 3G).

**Figure 3:** Steatohepatitis and sarcopenic obesity were induced by 20 weeks HFD feeding. 8-week-old and 42-week-old male C57BL/6 mice were fed with a HFD for 20 weeks, mice were sacrificed after the assessment of body composition and muscle strength, and liver and muscle tissues were harvested. **(A)** Representative hematoxylin and eosin staining of liver sections in mice (*n* = 6–9) are shown (scale bar, 50 μm), **(B)** NAFLD activity score based on the NAS score algorithm was measured (*n* = 6–9). **(C)** Body weights and **(D)** liver indexes of mice were weighed and calculated (*n* = 6–9). **(E)** Fat mass, fat mass/ bodyweight (BW), **(F)** lean mass/BW were measured using NMR (*n* = 5–8). **(G)** Grip strength was tested in *vivo* (*n* = 6–10). The data are presented as the mean ± SEM, unpaired two-tailed Student's *t*-test. *P < 0.05, ***P < 0.001, ****P < 0.0001.

### Twenty Weeks HFD Feeding Induced Muscle Weight and Histological Alterations

The change of muscle weight in HFD-fed young mice at week 20 was different from week 12. Specifically, quadriceps weight and proportion of HFD-fed group were no longer smaller than chow-fed group in young mice (Figures 4A,C). Moreover, the weight and proportion of gastrocnemius even exhibited a slight increasing trend in HFD-fed young mice (Figures 4B,D). HE staining of skeletal muscles revealed that HFD increased the gap between muscle fibers and decreased the mean muscle fiber diameter throughout the different age groups (Figures 4E,F). In addition, the Oil Red O staining of quadriceps in HFD-fed young mice did not exhibit a significant increase in the abundance of lipid droplets (Supplementary Figure 2A).

The article "Ammonia Scavenger Restores Liver and Muscle Injury in a Mouse Model of Non-alcoholic Steatohepatitis With Sarcopenic Obesity" was retracted in 2025. Reasons: plagiarism; overlap with other authors' work.

**Figure 4:** Muscle weight and histological changes of mice fed with HFD for 20 weeks. **(A)** Quadriceps and **(B)** gastrocnemius muscle weight are measured (*n* = 6–10). **(C)** Quadriceps weight and **(D)** gastrocnemius weight to body weight ratio are calculated (*n* = 6–10). **(E)** Representative hematoxylin and eosin staining pictures of quadriceps in mice (*n* = 5–10) are shown (scale bar, 50 μm). **(F)** Average myofiber diameters were quantified (*n* = 5–10). The data are presented as the mean ± SEM, unpaired two-tailed Student's *t*-test. *P < 0.05, **P < 0.01.

### HFD-Induced Hyperammonemia Was Associated With the Decline of Muscle Quality

In order to determine whether hyperammonemia will develop in NASH and explore the association between ammonia level and muscle phenotypes, we measured plasma ammonia level of mice at different time points (i.e., young mice at 4, 8, 12, and 20 weeks). Even though the plasma ammonia level of HFD-fed group was maintained at a relative low level at 8 and 12 weeks, it was always higher than that of chow-fed group (Figure 5A). At the end of the 20th week, the plasma ammonia concentration of HFD-fed group was dramatically increased and significantly higher than the chow-fed controls (Figure 5A). We also measured plasma ammonia levels of middle-aged mice at 20 weeks. Similarly, plasma ammonia levels were also significantly increased in the group of HFD-fed middle-aged mice (Figure 5B). When we carried out the correlation analysis for young mice at week 20, we found that plasma ammonia level showed a significant positive correlation with body weight, liver index, and NAS score, and a significant negative correlation with grip strength, and muscle fiber diameter (Figure 5C). However, no correlation was found between plasma ammonia level and body composition in young mice. Plasma ammonia levels of middle-aged mice was significantly positively correlated with liver index and NAS score, and negatively with muscle fiber diameter (Supplementary Figure 3A).

**Figure 5:** Correlation analysis between plasma ammonia level and other indexes in mice. **(A)** Plasma ammonia levels of young mice over the course of the experiment (*n* = 5–9). **(B)** The plasma ammonia level of young mice and middle-aged mice at the end of the 20th week is detected (*n* = 5–9). **(C)** Correlation between plasma ammonia level and other indexes in young mice including body weight, liver index, NAS score, fat mass, fat mass/bodyweight (BW), lean mass/BW, grip strength, and muscle fiber diameter (Spearman correlation analysis, *n* = 14–15). The data are presented as the mean ± SEM, unpaired two-tailed Student's *t*-test. *P < 0.05, **P < 0.01, ***P < 0.001.

The article "Ammonia Scavenger Restores Liver and Muscle Injury in a Mouse Model of Non-alcoholic Steatohepatitis With Sarcopenic Obesity" was retracted in 2025. Reasons: plagiarism; overlap with other authors' work.

### Hepatic Inflammation and Fibrosis Were Attenuated by LOLA in Mice Fed an HFD

We next assessed the effect of LOLA on liver injury induced by HFD feeding. In HFD-fed group, LOLA-treated mice have lower plasma ammonia levels than vehicle-treated mice (Figure 6A). Meanwhile, plasma levels of ALT, AST, and cholesterol were greatly elevated in mice fed an HFD and significantly declined with LOLA intervention (Figure 6A). Then, we performed HE staining to evaluate liver histology of mice. In contrast to vehicle-treated controls, HFD mice with LOLA treatment had greatly reduced lipid droplets and inflammatory foci in the liver, and significantly decreased NAS score (Figures 6C,D). Although the effect of LOLA on steatosis score and expression levels of hepatic lipid metabolism-related genes was not significant (Supplementary Figures 4A,D), lipid quantification results demonstrated that LOLA can reduce liver fat content with a decrease in triglyceride and cholesterol levels (Figure 6B). In addition to steatosis, we found the inflammation score and ballooning score in HFD-fed mice were significantly decreased by LOLA (Supplementary Figures 4B,C). Given that result, we examined the infiltration of inflammatory cells using immunohistochemical staining of their specific markers. Macrophages (labeled by F4/80 or CD68), especially Kupffer cells, which were considered as the key mediator of hepatic inflammation during NASH development (24, 25), were decreased by LOLA compared with those in vehicle-treated group (Figures 6C,F). Neutrophils (labeled by MPO), another important inflammatory cell, were also significantly reduced in the hepatic lobule of mice with LOLA intervention (Figures 6C,E). Correspondingly, hepatic expression of inflammation-related genes (TNFα, IL6, CCL2, CCR2) was significantly increased in HFD-fed mice and decreased with LOLA treatment (Supplementary Figure 4E). Moreover, we determined whether LOLA has a protective effect on HFD-induced liver fibrosis. Sirius red staining and qPCR results demonstrated that LOLA significantly reduced hepatic collagen deposition and inhibited the mRNA expression of fibrosis-related genes (αSMA, TGFβ, Col1α1, Col1α2) in mice fed an HFD (Figures 6C,G; Supplementary Figure 4F). Immunolocalization of αSMA, a stellate cell proliferation marker (26), was decreased in LOLA-treated group compared with vehicle-treated controls, suggesting a marked decrease in fibrosis and stellate cell proliferation (Figures 6C,G).

The article "Ammonia Scavenger Restores Liver and Muscle Injury in a Mouse Model of Non-alcoholic Steatohepatitis With Sarcopenic Obesity" was retracted in 2025. Reasons: plagiarism; overlap with other authors' work.

**Figure 6:** LOLA attenuates HFD-induced liver injuries. Eight-week-old male C57BL/6 mice were fed with a HFD for 12 weeks, and then gavaged with L-ornithine L-aspartate (LOLA) (2 g/kg/day) or vehicle (0.9% saline) for 8 weeks. Mice were sacrificed after the assessment of body composition and muscle strength, then liver and muscle tissues were harvested. **(A)** Plasma levels of ammonia, Alanine aminotransaminase (ALT), aspartate aminotransaminase (AST), and cholesterol are measured (*n* = 6). **(B)** Hepatic triglyceride levels and cholesterol levels are assessed in mice (*n* = 6). **(C)** Representative pictures of hepatic hematoxylin and eosin staining, immunohistochemical staining of F4/80, myeloperoxidase (MPO), CD68, alpha-smooth muscle actin (αSMA), and Sirius Red staining (*n* = 6) are shown (scale bars, 50 μm). **(D)** NAFLD activity score based on the NAS score algorithm was measured (*n* = 6). **(E)** Quantification of MPO, **(F)** F4/80 and CD68 positive cells expressed as a percentage of those in the HFD-fed vehicle-treated group (*n* = 4–10). **(G)** Quantification of Sirius Red and αSMA are shown (*n* = 4–10). The data are presented as the mean ± SEM, unpaired two-tailed Student's *t*-test. *P < 0.05, vs. mice fed with chow diet; ^#^*P* < 0.05, vs. mice fed with high-fat diet.

### Ammonia Lowering Improved HFD-Induced Sarcopenic Obesity in Mice

Eight-week LOLA intervention did not alter body weight of HFD-fed mice (Figure 7A). However, body composition was markedly changed in mice received LOLA gavage. Fat mass and percentage body fat were significantly decreased in LOLA-treated mice while lean body mass was significantly increased compared with the vehicle-treated controls (Figures 7B,C). Meanwhile, LOLA significantly restored HFD-induced decline in muscle strength (Figure 7D). The average myofiber diameter was higher in quadriceps of LOLA-treated mice compared with vehicle-treated controls, as evidence by HE staining (Figures 7E,F). The above results suggest that LOLA has a beneficial role in protecting muscle quality.

**Figure 7:** LOLA improved sarcopenic obesity in mice fed with an HFD. **(A)** Body weight of mice after LOLA intervention are measured (*n* = 8–10). **(B)** Fat mass, fat mass/bodyweight (BW), **(C)** lean mass/BW are detected by NMR (*n* = 6). **(D)** Forelimb grip strength is tested (*n* = 6). **(E)** Representative hematoxylin and eosin staining pictures of quadriceps in mice (*n* = 6) are shown (scale bar, 50 μm). **(F)** Mean diameters of muscle fibers are quantified (*n* = 6). The data are presented as the mean ± SEM, unpaired two-tailed Student's *t*-test. *P < 0.05, vs. mice fed with chow diet; ^#^*P* < 0.05, vs. mice fed with HFD.

The article "Ammonia Scavenger Restores Liver and Muscle Injury in a Mouse Model of Non-alcoholic Steatohepatitis With Sarcopenic Obesity" was retracted in 2025. Reasons: plagiarism; overlap with other authors' work.

## Discussion

This study used an HFD to feed mice at different ages and dynamically observed the changes in body composition, liver, and muscle lesions. Our results showed that long-term HFD feeding could successfully induce a mouse model that contains the phenotype of both NASH and sarcopenic obesity. Besides, the onset of steatohepatitis was earlier than sarcopenia in this model. The high blood ammonia level caused by hepatic dysfunction might be an important factor in promoting the development of sarcopenia in mice. Ammonia lowering drug LOLA showed a significant efficacy in the treatment of steatohepatitis and sarcopenia.

In recent years, the complex relationship between NAFLD and skeletal muscle disorders has become a focus of clinical attention. A better understanding of the pathogenesis and natural course of sarcopenia in NAFLD may help to improve the diagnosis and treatment of these two diseases. The HFD-induced model is a commonly used NASH model, while less attention has been given to the muscle status in NASH mice. Given that age is an essential factor influencing muscle health, we performed the same experiments in both young and middle-aged mice. After 20 weeks of modeling, all mice in the HFD group developed not only NASH but also sarcopenic obesity. Although there were no significant changes in body weight of these mice, they exhibited increased body fat mass and significant muscle loss, which are similar to the features of non-obese NAFLD. Normally, a significant proportion of non-obese NAFLD patients have high body fat content or abdominal obesity (2, 27), whereas their muscle mass is relatively lower than obese patients and healthy individuals. Thus, the BMI-based typing system cannot fully reflect the status of obesity in NAFLD, and it should be replaced by some precise methods such as body composition analysis to find patients with NAFLD complicated by occult obesity and sarcopenia. Taken together, this diet-induced NASH model is simple, easy to perform, and has high success rate, which could be used for studies of non-obese NAFLD pathogenesis and new drug research and development.

Series of clinical studies have revealed that NAFLD and sarcopenia have several identical pathophysiological mechanisms and mutually promote the development of each other (28, 29), but they failed to draw conclusions about the cause-and-effect relationships among them. To investigate this question, we detected muscle mass and function of NASH mice at two different time points, in which 12 weeks represents the early stage of NASH and 20 weeks represents the advanced stage of NASH. We observed that young mice manifested only declined muscle strength in the early stage of NASH, and they met the working definition of sarcopenia until the late phase. Our results suggest that sarcopenia presents later than NASH. It is more like a consequence or a complication in the development of NAFLD. This result is consistent with the recent finding that only fibrosing NASH is associated with sarcopenia among the NAFLD spectrum (30). Results from the middle-aged group suggest that the older mice could have more severe steatohepatitis and sarcopenia comparing with younger mice over the same period. Aging is a well-known cause of sarcopenia. Several factors that accompany senescence, including altered hormone levels and low activity, will inevitably exacerbate the decline of muscle mass and quality (31). This hints that clinical workers should pay more attention to the muscle health of old NAFLD patients.

The article "Ammonia Scavenger Restores Liver and Muscle Injury in a Mouse Model of Non-alcoholic Steatohepatitis With Sarcopenic Obesity" was retracted in 2025. Reasons: plagiarism; overlap with other authors' work.

Another interesting finding of this study is that the muscle weight in HFD-fed mice changed with the time duration of the study. In the early stage of NASH, HFD-fed young mice showed relatively low muscle weight than chow-fed controls. However, muscle weight was similar in the two groups at the end of the experiment. We observed that mice in the HFD group were less active during the experiment, which could be one of the reasons for the initial reduction of muscle weight. Besides liver steatosis, the HFD may also induce ectopic fat deposition in muscle tissues which is so-called myosteatosis. Recent study has reported that myosteatosis could present in both early and fibrosing NASH, and its degree has a strong correlation with liver disease activity (30). Thus, we speculate that the long-term HFD feeding might lead to a rebound in muscle weight by inducing myosteatosis.

The pathogenesis of sarcopenia in NAFLD patients is not yet clear. Our data suggest that steatohepatitis-induced hyperammonemia may play a role in the development of sarcopenia. Normally, ~50% of the arterial ammonia was metabolized by skeletal muscle, and muscle may become the most important organ for ammonia detoxification when patients have serious liver dysfunction (32). However, since ammonia has an adverse impact on bioenergetics and protein homeostasis of muscles (15), increased ammonia uptake into muscle will inevitably lead to muscle damage. In agreement with the previous study (17), we found that blood ammonia level was significantly elevated in NASH mice. Moreover, there was an inverse correlation between ammonia concentration and grip strength in young mice. This finding motivated our speculation that ammonia lowering may have beneficial effects on protecting muscles in NASH mice.

The article "Ammonia Scavenger Restores Liver and Muscle Injury in a Mouse Model of Non-alcoholic Steatohepatitis With Sarcopenic Obesity" was retracted in 2025. Reasons: plagiarism; overlap with other authors' work.

LOLA has been recognized as an effective ammonia-lowering drug for several years with good evidence in hepatic encephalopathy, and it also showed a protective effect of skeletal muscle proteostasis in a rat model of liver cirrhosis (33, 34). Our *in vivo* results showed that LOLA treatment can reduce plasma ammonia and restore muscle mass and strength in mice with an HFD. Besides improving muscle health, our results revealed that LOLA also has great efficacy in liver injuries, especially hepatic inflammation and liver fibrosis. As a toxic metabolite, ammonia affects various organs and tissues within the body. Some studies have reported that ammonia can fuel activation of hepatic stellate cells and liver fibrosis and ammonia scavenger can effectively prevent the progression of NASH to fibrosis (17, 35). These results highlight the therapeutic potential of LOLA in NASH and sarcopenia management.

There are several limitations to this study. Firstly, we did not find the evidence of worsened myosteatosis in HFD mice. One possible reason is that oil red o staining is not sufficiently sensitive to evaluate muscle fat deposition. Instead, computed tomography (CT) and MRI as the gold standards for assessing muscle quality are more suitable for the detection of myosteatosis (22). Another possible reason is that the degree of myosteatosis might be varied in different muscle tissues. Compared with measuring thigh muscles, clinical studies generally prefer to choose dorsal muscles such as psoas muscles and paraspinous muscles at L3 or L4 levels as examination sites for muscle quality (36, 37). Hence, it is possible that if we had selected a sensitive technique or examined muscles in other parts of the body, we would have observed some different results regarding myosteatosis. Secondly, it is a pity that we did not set more observation points between week 12 and week 20 to catch the key timepoint at which plasma ammonia augmentation was initiated. Moreover, whether high blood ammonia level could directly exacerbate liver and muscle injury in NASH mice need further experimental confirmation.

In conclusion, the current study establishes a rodent model of steatohepatitis with sarcopenia that provides good experimental material for research on non-obese NAFLD, and provides a clue that ammonia lowering could be a promising therapeutic strategy for sarcopenia in patients with liver disease. The efficacy of LOLA on NASH and sarcopenia needs to be validated in a large cohort of patients. Ongoing work in our laboratory is seeking to answer these questions.

The article "Ammonia Scavenger Restores Liver and Muscle Injury in a Mouse Model of Non-alcoholic Steatohepatitis With Sarcopenic Obesity" was retracted in 2025. Reasons: plagiarism; overlap with other authors' work.

## Data Availability Statement

The original contributions presented in the study are publicly available. This data can be found here: https://www.jianguoyun.com/p/Df66hEAQ5KL_CRj1yZgE / code: 6D0u7z.

## Ethics Statement

The animal study was reviewed and approved by Institutional Animal Care and Use Committee of Xinhua Hospital Affiliated to Shanghai Jiao Tong University School of Medicine.

## Author Contributions

Z-XW, J-GF, and YL contributed to the experiment design. Z-XW, M-YW, R-XY, Z-HZ, F-ZX, and T-YR contributed to the acquisition and analysis of data. J-GF and R-XY obtained the funding. Z-XW and M-YW wrote the article. J-GF, T-YR, and R-XY revised the article. All authors contributed to the article and approved the submitted version.

## Funding

This work was supported by National Natural Science Foundation of China (81873565 and 82170593), Shanghai Leading Talent Plan 2017, Star Program of Shanghai Jiaotong University (YF2021QN54), and Hospital Funded Clinical Research, Clinical Research Unit, Xinhua Hospital Affiliated to Shanghai Jiao Tong University School of Medicine (17CSK04) to J-GF. This work was also supported by grants from National Natural Science Foundation of China (81900507) to R-XY and (82100606) to T-YR.

## Conflict of Interest

The authors declare that the research was conducted in the absence of any commercial or financial relationships that could be construed as a potential conflict of interest.

## Publisher's Note

All claims expressed in this article are solely those of the authors and do not necessarily represent those of their affiliated organizations, or those of the publisher, the editors and the reviewers. Any product that may be evaluated in this article, or claim that may be made by its manufacturer, is not guaranteed or endorsed by the publisher.

## Supplementary Material

Supplementary Figure 1 The scheme of animal experiments. **(A)** The flow diagram of establishing the mouse model of steatohepatitis with sarcopenic obesity. **(B)** The flow diagram of administration of LOLA.

Supplementary Figure 2 Muscle fat infiltration in young mice at week 20. The representative pictures of oil red o staining for quadriceps in young mice (*n* = 3) at the end of the 20th week are shown (scale bar, 50 μm).

Supplementary Figure 3 The correlation analysis of plasma ammonia and other indexes in middle-aged mice at week 20. **(A)** Correlation between plasma ammonia level and other indexes in middle-aged mice including body weight, liver index, NAS score, fat mass, fat mass/BW, lean mass/BW, grip strength, and muscle fiber diameter (Spearman correlation analysis, *n* = 10–11). The data are presented as the mean ± SEM.

The article "Ammonia Scavenger Restores Liver and Muscle Injury in a Mouse Model of Non-alcoholic Steatohepatitis With Sarcopenic Obesity" was retracted in 2025. Reasons: plagiarism; overlap with other authors' work.

Supplementary Figure 4 Detailed NAFLD activity score and hepatic gene expression analysis in mice treated with LOLA. **(A)** Steatosis score, **(B)** inflammation score, and **(C)** ballooning score based on the NAS scoring system are evaluated (*n* = 6). The expression levels of **(D)** lipid metabolism-related genes (SREBP1c, FAS, SCD1, PPARα, and CPT1A), **(E)** inflammation-related genes (TNFα, IL6, CCL2, CCR2), and **(F)** fibrosis-related genes (αSMA, TGFβ, Col1α1, Col1α2) are determined by real-time PCR. Relative expression levels were normalized to those of actin. The data are presented as the mean ± SEM, unpaired two-tailed Student's *t*-test. **P* < 0.05, vs. mice fed with chow diet; ^#^*P* < 0.05, vs. mice fed with HFD.
